The article "Effects of Short- and Long-Term Detraining on Maximal Oxygen Uptake in Athletes: A Systematic Review and Meta-Analysis" was published in 2022. Journal: Biomed Res Int.

# Effects of Short- and Long-Term Detraining on Maximal Oxygen Uptake in Athletes: A Systematic Review and Meta-Analysis

**DOI:** 10.1155/2022/2130993

**Published:** 2022-08-16

**Authors:** Jie Zheng, Tian Pan, Yankang Jiang, Yupeng Shen

**Affiliations:** School of Physical Education and Sports Science, South China Normal University, Guangzhou 51000, China

## Abstract

V̇O_2_max, a gold standard for evaluating cardiorespiratory fitness, can be enhanced by training and will gradually decrease when training stops. This study, which followed the Cochrane Collaboration guidelines, is aimed at assessing the effect of short- and long-term detraining on trained individuals' V̇O_2_max through a systematic review and meta-analysis and performed a subgroup analysis to evaluate the effects of different ages, detraining formats, and training statuses on V̇O_2_max variation between short- and long-term training cessation. Web of Science, SPORTDiscus, PubMed, and Scopus, four databases, were searched, from which 21 of 3315 potential studies met the inclusion criteria. Significant decreases in V̇O_2_max were identified after short-term training cessation (ES = −0.62 [95% CI -0.94; -0.31], *p* < 0.01; within-group *I*^2^ = 35.3%, Egger′s test = −1.22, *p* = 0.335) and long-term training cessation (ES = −1.42 [95% CI -1.99; -0.84], *p* < 0.01; within-group *I*^2^ = 76.3%, Egger′s test = −3.369, *p* < 0.01), which shows that the detraining effect was found to be larger on V̇O_2_max in long-term training cessation than in short-term training cessation (*Q* = 6.5, *p* = 0.01). However, there was no significant difference regarding V̇O_2_max change between 30-90 days detraining and larger than 90 days detraining (*Q* = 0.54, *p* = 0.46) when conducting subgroup analysis. In addition, younger (<20) individuals showed a greater reduction in V̇O_2_max after long-term detraining than adult individuals (*Q* = 5.9, *p* = 0.05), and athletes with higher trained-state V̇O_2_max showed a significant decline in V̇O_2_max after long-term detraining compared with the lower trained-state group (*Q* = 4.24, *p* = 0.03). In conclusion, both short- and long-term training cessation have a detrimental effect on V̇O_2_max, and a greater impact on V̇O_2_max was found in long-term training cessation compared to short-term training cessation; however, there was no significant change in V̇O_2_max when the duration of training cessation was more than 30 days. To buffer the detrimental effects of detraining, especially long-term training cessation, performing some physical exercise during training cessation can effectively weaken detraining effects. Thus, to prevent athlete's V̇O_2_max from decreasing dramatically from detraining, athletes should continue performing some physical exercise during the cessation of training.

The article "Effects of Short- and Long-Term Detraining on Maximal Oxygen Uptake in Athletes: A Systematic Review and Meta-Analysis" was published in 2022. Journal: Biomed Res Int.

## 1. Introduction

Maximal oxygen uptake (V̇O_2_max) is defined as the maximal rate at which oxygen can be taken up and utilized by the body during high-intensity exercise. Generally, V̇O_2_max is considered the most effective tool to measure the functionality of the human cardiovascular system [1, 2] and an effective indicator to explain individual cardiorespiratory health [3]. In addition, V̇O_2_max is a determinant of endurance performance for athletes [4] and one of the standard methods to evaluate the effects of aerobic training on athletes. Sports training and physical exercise are effective means to improve and maintain V̇O_2_max and have been widely verified in healthy [5], obese or overweight [6, 7], and athlete populations [8, 9]. However, the adaptability of V̇O_2_max obtained through training is reversible. It will diminish when the training stimulus disappears or decreases significantly [10]. The cessation of training reduces or removes the training stimulus and leads to the loss of anatomical, physiological, and performance training adaptability, which is defined as a detraining effect. The detraining effect on V̇O_2_max was related to the periods of training cessation, and the duration of the training cessation can be categorized as a short-term (less than four weeks) or long-term (more than four weeks) period in a previous study [10, 11]. Mujika and Padilla [10, 11] summarized some research findings that V̇O_2_max for highly trained athletes decreased by 4-14% after short-term detraining but decreased by 6-20% after long-term detraining. Although long-term detraining seems to have a greater impact on V̇O_2_max than short-term detraining, the lack of effective comparison methods makes it unclear how the detraining length affects athletes' V̇O_2_max.

The high V̇O_2_max level results from long-term regular exercise to benefit the cardiovascular circulatory system and muscle function. Some studies have reported that V̇O_2_max in trained people can remain unchanged after short-term detraining [12]. However, another study has shown that a higher V̇O_2_max training status results in a greater decrease in V̇O_2_max after short-term detraining [10]. The level of V̇O_2_max in highly trained athletes initially decreases progressively, but eventually, V̇O_2_max can be maintained at the control level after the long-term period [11], while those without an untrained background will completely lose their V̇O_2_max gain after a long-term period. These studies indicated that the training status of V̇O_2_max before detraining might affect the adverse effects of training cessation on V̇O_2_max between short- and long-term periods. Nevertheless, limited research makes the influence of V̇O_2_max training status on the relationship between the duration of training cessation and V̇O_2_max in trained athletes still controversial.

The article "Effects of Short- and Long-Term Detraining on Maximal Oxygen Uptake in Athletes: A Systematic Review and Meta-Analysis" was published in 2022. Journal: Biomed Res Int.

When exposed to the risk of detraining, athletes will face two forms of detraining: one is complete cessation of training (CDT), that is, in addition to daily physical activity, complete interruption of training; the other is partial cessation of training (PDT), that is, doing exercise at a certain intensity of each week during detraining [10, 13]. Compared with CDT, PDT seems to reduce or offset the adverse effects on physiological functions and morphology. A recent study has shown that the losses in training adaptations and exercise capacity that occur during periods of inactivity may at least be partially alleviated with a program of reduced training frequency and/or duration if intensity is maintained [14]. Barry et al. [12] reported that conducting a 40-minute training program at 80% HRmax intensity twice a week can maintain V̇O_2_max for the general population until 15 weeks. For the athlete group, research by Houmard and Mujika and Padilla [13, 15, 16] showed that the training frequency needs to be maintained above 80% of the original to decrease endurance performance. Although PDT is a training strategy to reduce the adverse effects of detraining, athletes have a different physiological response to training cessation in the short term or long term. Compared with CPT, the benefit and validation of PDT have not been evaluated by systematic review.

Changes in V̇O_2_max and endurance performance are related to age. Endurance performance can show the highest level only after 20 [17], and V̇O_2_max in adolescents is lower than that of adults because V̇O_2_max can reach the peak level after 20 years of age [18]. V̇O_2_max reflects muscles' ability to utilize oxygen. Lemmer et al. confirmed that the strength retention rate of young people is significantly greater than that of elderly people after 12-31 weeks of training cessation [18]. Although these studies may imply that age may play a moderating role in detraining V̇O_2_max, no studies have evaluated the effect of detraining V̇O_2_max between the adolescent population (<20) and adults (≥20).

Recently, the COVID-19 outbreak has exposed athletes to the risk of detraining, which dramatically raises the possibility of a decline in athletic performance, the disappearance of training adaptation, and the risk of injury. It is an emerging challenge for athletes and coaches to formulate appropriate detraining prevention strategies, which require us to comprehend the effect of detraining on V̇O_2_max. Nevertheless, the relevant assessment will be limited by different research methods. High-quality systematic reviews and meta-analyses can help us overcome these challenges, explain the bias and homogeneity of these studies, and provide a more accurate assessment of the effects. Therefore, the purpose of this study is to evaluate the impact of short- and long-term detraining on V̇O_2_max and assess the effects of age, training status, and detraining format on V̇O_2_max between the long- and short-term periods by a subgroup analysis.

The article "Effects of Short- and Long-Term Detraining on Maximal Oxygen Uptake in Athletes: A Systematic Review and Meta-Analysis" was published in 2022. Journal: Biomed Res Int.

## 2. Materials and Methods

This systematic review and meta-analysis followed the Cochrane Collaboration guidelines [19]. The systematic review strategy was conducted according to PRISMA (Preferred Reporting Items for Systematic Reviews and Meta-analyses) guidelines [20].

The literature search, identification, screening, and data extraction were conducted independently by two reviewers (TP and JZ). Disagreements between the reviewers were resolved by consensus or arbitration through a third reviewer (YkJ). Papers that were clearly not relevant were removed from the database list before abstracts were assessed using predetermined inclusion and exclusion criteria. The process of the study selection is shown in Figure 1.

### 2.1. Search Strategy

Electronic databases were searched in Web of Science, SPORTDiscus, PubMed, and Scopus. Searches were limited to papers published in English and from relevant publications prior to 31 March 2021. Keywords and synonyms were entered in various combinations (detraining OR deconditioning OR “training cessation” AND endurance^∗^ OR lactate^∗^ OR V̇O_2_max OR aerobic^∗^).

### 2.2. Selection Criteria

Studies were eligible for inclusion if (a) the paper reported a specific detraining duration and gave a detailed value of V̇O_2_max before and after detraining, (b) the research subjects were athletes and were not limited by age, sex, event, or competitive level, and (c) articles were written in English.

Studies were excluded if (a) the paper reported relevant information unclearly or (b) the full text could not be obtained.

### 2.3. Extraction of Data

The characteristics of the 21 studies included in the meta-analysis can be found in Table 1. Two independent reviewers (TP and JZ) read and coded each included study using the following moderators: authors and year of publication; training status (higher or lower); duration (days); sex (male, female, or mixed); age (<20 or ≥20); and detraining format (CDT or PDT).

### 2.4. Quality Assessment

Table 2 presents the summary of the STROBE statement checklist. The quality assessment was conducted independently by two reviewers (JZ and YkJ), and disagreements about outcomes were resolved by consensus or arbitration through a third reviewer (TP). The included articles were conducted using the Strengthening the Reporting of Observational studies in Epidemiology (STROBE) checklist for cohort studies [21]. This checklist scores 22 items in the categories of title and abstract (item 1), introduction (items 2-3), methods (items 4-12), the results (items 13-17), discussion (items 18-21), and other information (item 22).

The article "Effects of Short- and Long-Term Detraining on Maximal Oxygen Uptake in Athletes: A Systematic Review and Meta-Analysis" was published in 2022. Journal: Biomed Res Int.

### 2.5. Synthesis of Results

Meta-analyses were conducted by the Meta package in R Studio (v1.41, Boston, USA). When comparing the duration of detraining effects on V̇O_2_max, the outcome data were divided into short-term (≤30 days) and long-term (>30 days) [10], and long-term periods of detraining were organized into 30-90 days and >90 days for further analysis in the long-term detraining period [11]. The standardized mean difference (SMD) for each study was calculated as Hedge's g effect size (ES) [22] to evaluate the magnitude of effects in different studies. Cohen's criteria [23] were used to interpret the magnitude of SMD: <0.5, small; 0.5 to 0.8, moderate; and >0.8, large. Data are presented as the mean and 95% CI. *I*^2^ is used to quantify statistical heterogeneity as follows [24]: 0% to 40%: might not be important; 30% to 60%: may represent moderate heterogeneity^∗^; 50% to 90%: may represent substantial heterogeneity^∗^; and 75% to 100%: considerable heterogeneity^∗^ [25]. A fixed model was used for analysis; however, if statistical heterogeneity was shown (*I*^2^ < 40%), meta-analyses were performed using a random-effects model. Extended Egger's test [26] was used to assess the risk of bias across the studies.

## 3. Results

### 3.1. Study Identification and Selection

The search of databases and additional titles from other sources identified an initial 3315 titles. These studies were then exported to reference manager software (EndNoteX9, USA). Duplicates (1865 references) were subsequently removed either automatically or manually. The remaining 1450 articles were screened for their relevance based on titles and abstracts, resulting in the removal of an additional 1271 studies. The full texts of the remaining 179 articles were examined diligently; 158 articles were rejected as they did not satisfy the relevant criteria, including the following: full text could not be obtained (*n* = 32); studies did not report specific data (*n* = 6); nonathletes (*n* = 51); training (*n* = 18); unrelated (*n* = 25); and others (*n* = 26). Twenty-one articles were eligible for the systematic review and meta-analysis (Figure 1). The 21 studies included provided mean and standard deviation V̇O_2_max data for at least one main outcome.

The article "Effects of Short- and Long-Term Detraining on Maximal Oxygen Uptake in Athletes: A Systematic Review and Meta-Analysis" was published in 2022. Journal: Biomed Res Int.

### 3.2. Study Characteristics

The characteristics of the 21 studies included in the meta-analysis can be found in Table 1. Detraining periods varied between 10 and 730 days across the studies. Twenty-one studies were divided into short-term (<30 days), long-term (30-90 days), and ultralong-term (>90 days) studies.

Table 2 presents the summary of the STROBE statement checklist. From the 21 included studies in the meta-analysis, five studies were classified between 28 and 31, eleven between 32 and 35, and five between 36 and 39.

### 3.3. The Effects of Short-Term and Long-Term Training Cessation on V̇O_2_max

The forest plot shows the effects of short-term and long-term detraining on V̇O_2_max. Significant decreases in V̇O_2_max were identified after short-term training cessation (ES = −0.62 [95% CI -0.94; -0.31], *p* < 0.01; within-group *I*^2^ = 35.3%, Egger′s test = −1.22, *p* = 0.335) and long-term training cessation (ES = −1.42 [95% CI -1.99; -0.84], *p* < 0.01; within-group *I*^2^ = 77%, Egger′s test = −3.369, *p* < 0.01). The detrimental effect of detraining was found to be larger in long-term training cessation than in short-term training cessation (*Q* = 6.5, *p* = 0.01). The relative weight of each study in the short-term training cessation and long-term training cessation varied between 2.8% and 3.1% and between 1.6% and 3.6%, respectively (Figure 2).

### 3.4. Subgroup Analysis Results

The effect of training cessation on V̇O_2_max after long-term detraining is presented in Table 3. The subgroup analysis showed that there was no significant difference regarding V̇O_2_max change between 30-90 days detraining and larger than 90 days detraining (*Q* = 0.54, *p* = 0.46). However, the athletes with higher trained-state V̇O_2_max had a significant decline in V̇O_2_max after long-term detraining compared with the athletes with lower trained-state V̇O_2_max (*Q* = 4.24, *p* = 0.03). Younger (<20) trained individuals showed a greater reduction in V̇O_2_max after detraining than adult (≥20) trained individuals (*Q* = 5.9, *p* = 0.05). Compared with CDT, PDT had smaller effects of training cessation on V̇O_2_max (*Q* = 6.23, *p* = 0.01). The short-term detraining effect on V̇O_2_max is shown in Table 4. For short-term training cessation, the effect of detraining was not changed significantly between higher and lower trained-state V̇O_2_max athletes (*Q* = 1.45, *p* = 0.22), between ages (*Q* = 0.27, *p* = 0.87), or between CDT and PDT (*Q* = 0.36, *p* = 0.55).

## 4. Discussion

This systematic review and meta-analysis is aimed at assessing the magnitude of the effect on trained individuals' V̇O_2_max after short- and long-term training cessation. A detrimental impact on trained individuals' V̇O_2_max was observed during both short- and long-term training cessation, and a larger negative effect after the long-term period was identified compared with the short-term period. The subgroup analysis showed that the effects of age, training status, and detraining format led to the differing impacts of detraining on V̇O_2_max in the long-term period but did not change in the short-term period.

The article "Effects of Short- and Long-Term Detraining on Maximal Oxygen Uptake in Athletes: A Systematic Review and Meta-Analysis" was published in 2022. Journal: Biomed Res Int.

### 4.1. The Short-Term and Long-Term Effects on V̇O_2_max

The present study revealed that both short- and long-term detraining will cause a significant drop in the trained individual's V̇O_2_max, and the average V̇O_2_max decreased by 3.93% in the short-term period and by 9.43% in the long-term period. Training cessation or reduction causes insufficient or disappearance of training stimulation and leads to morphological and physiological functional changes, which may be the main factor for the harmful effects of long-term and short-term detraining on V̇O_2_max [10, 11]. It is worth noting that there was no significant difference in the decline in V̇O_2_max between 30-90 days and longer than 90 days detraining in the subgroup analysis of long-term detraining. This result indicated that when training cessation occurred beyond a certain period, the harmful effects on V̇O_2_max no longer increased with the extension of the training suspension time. In fact, even without physical training, daily essential physical activity can also maintain normal physiological function and sustain cardiovascular fitness [48], which may help to explain the nonlinear relationship between the duration of training cessation and detraining effects in the long term. The research results show that there is a dose-effect relationship between the detraining duration and the detraining effect. When the training cessation exceeds a certain period (>90 days), the harmful effects caused by the training suspension will no longer continue to worsen. In practice, coaches and athletes must be aware of the difference between the short- and long-term harmful effects of V̇O_2_max to develop detraining prevention strategies. Long-term detraining needs to be avoided because long-term detraining has a greater detrimental effect on V̇O_2_max.

### 4.2. Detraining Format Differences in the Short-Term and Long-Term Effects on V̇O_2_max

An essential finding of this study is that exercise activities during long-term detraining can reduce the negative effect of detraining on V̇O_2_max compared with no exercise activities. However, there was no significant difference in the harmful effects of V̇O_2_max between CDT and PDT. The magnitude of detrimental impacts on V̇O_2_max in the PDT groups during the long-term period was small, and the percentage of decline in V̇O_2_max ranged from -4.38% to -0.93%; however, the negative effect was large, and V̇O_2_max decreased up to -11.12%. Recent research also supports the results of the current study and shows that performing jogging exercises with 50-60% V̇O_2_max intensity for 20-30 minutes each time 2-3 times a week during off-seasonal periods can offset the harmful effects of detraining on V̇O_2_max in football players [49, 50]. Many studies have shown that regular aerobic exercise can maintain a healthy level of V̇O_2_max in the human body [51–54]. This may be helpful to explain why athletes who exercise can delay the decline in oxygen uptake during long-term training cessation. It was unexpected that PDT had no buffering effect on the harmful impacts of V̇O_2_max during the short-term period. There were small negative effects on V̇O_2_max in both the CDT and PDT groups, and the decrease in V̇O_2_max levels of athletes ranged from -21.28% to 0.84% in the CDT group and varied from -4.38% to -0.93% in the PDT group. One possible explanation is that the intensity of the exercise is inappropriate. In the sample of this study, the exercise intensity during the short-term period was low, which may not play a role in maintaining V̇O_2_max. Recent studies have also shown that exercise intensity is the key for athletes to sustain V̇O_2_max [12]. It has been reported that high-intensity exercise 2 times a week can allow athletes to maintain V̇O_2_max for 15 weeks without decreasing [12]. In addition, there may be a minimum threshold for the reduction of V̇O_2_max during training cessation. In this study, a minimum of 2 weeks of training can cause a decrease in V̇O_2_max, and the research results suggest that athletes and coaches need to consider the different effects of long- and short-term detraining when making detraining prevention plans. During the long-term period, necessary exercise can offset some of the negative impacts on V̇O_2_max. In the short term, if there is not enough stimulation, there may be no difference in V̇O_2_max change between athletes who exercise and those who do not exercise at all.

The article "Effects of Short- and Long-Term Detraining on Maximal Oxygen Uptake in Athletes: A Systematic Review and Meta-Analysis" was published in 2022. Journal: Biomed Res Int.

### 4.3. The Training Status Difference in the Short-Term and Long-Term Effects on V̇O2max

Long-term detraining has a more significant negative impact on athletes with higher levels of oxygen uptake training, which may be related to the training intensity that affects aerobic capacity. Studies have shown that training intensity rather than training frequency is crucial in maintaining V̇O_2_max levels [1, 55]. Athletes with higher training levels rely on higher training intensity to improve their physiological functions. Once training stimulation is lost, the training-induced gain for V̇O_2_max cannot be maintained. Long-term detraining makes the V̇O_2_max gain obtained by athletes through high-intensity training decrease or disappear more quickly. Athletes with a higher training status of V̇O_2_max have a more significant reduction in V̇O_2_max. The effect of short-term training cessation on V̇O_2_max was not affected by the level of V̇O_2_max, and there was no significant difference between the high-level and low-level groups. The current study is inconsistent with previous studies. Mujika and Padilla [10] summarize the results of some studies that show that athletes with higher oxygen uptake or aerobic power capacity have a more significant decrease in V̇O_2_max ranging between 4 and 14% after short-term training stops. The differences in the results of different studies may be due to the limitations of the previous research methods. Although previous studies have reported a greater percentage drop rate for athletes with a higher training status of V̇O_2_max, this is not enough to cause a significant difference in the magnitude of an adverse effect of training suspension on V̇O_2_max.

### 4.4. The Age Difference in the Short-Term and Long-Term Effects on V̇O_2_max

After long-term training cessation, the changes in athletes' V̇O_2_max were affected by age. Compared with adult athletes, young athletes have a greater rate of decline in V̇O_2_max after long-term suspension. In general, V̇O_2_max can reach its peak level at the age of 20-30 and decreases by approximately 1% every year after 30 [56]. Therefore, a lack of long-term training stimulation may have a more significant impact on the cardiovascular function of young athletes than adult athletes. Only one study reported the effect of short-term training on V̇O_2_max for the adolescent population [35]. Therefore, it is impossible to examine the effect of age on V̇O_2_max during short-term training for subgroup analysis. Meanwhile, only three studies reported on V̇O_2_max for the junior [28, 35, 45] group, and the limited research samples required us to treat the study results with caution.

### 4.5. Research Limitations and Future Prospects

More research samples in this study come from male athletes or mixed genders, and only two studies are female athletes. The differences in the physiological structure of men and women [33] may affect the results of the study. It is necessary to examine the difference in V̇O_2_max change between sexes after short- and long-term detraining in subsequent studies. In addition, factors such as nutrition (i.e., sports supplementation), environment, or measurement methods may affect the changes in oxygen uptake during detraining [57–61]. Therefore, the effects of these factors on the change in oxygen uptake during training cessation will also be considered in a follow-up study. Studies have shown that certain exercises can buffer some harmful effects during long-term periods, but current research cannot identify the training intensity and training load of certain exercises. In future research, it is necessary to explore the minimum dose-effect relationship that can maintain V̇O_2_max after detraining. Previous studies have reported that V̇O_2_max is related to changes in physical fitness levels, and future studies should compare the differences in physical fitness. Finally, research bias may have affected the research results.

The article "Effects of Short- and Long-Term Detraining on Maximal Oxygen Uptake in Athletes: A Systematic Review and Meta-Analysis" was published in 2022. Journal: Biomed Res Int.

## 5. Conclusion

The detrimental effects of detraining on V̇O_2_max were identified in both short-term and long-term training cessation. A greater decline in V̇O_2_max after the long-term period was observed when it was compared to short-term training cessation; however, there was no significant difference regarding the reduction in V̇O_2_max found between 30-90 days detraining and more than 90 days detraining. Physical exercise during the period of detraining seems to weaken the detrimental effects on V̇O_2_max to some extent during long-term training cessation, but it does not work in short-term training cessation. Adolescent and individual trainers with a higher V̇O_2_max training status have a greater decline in oxygen uptake after long-term training cessation.

## Figures and Tables

**Figure 1:** Flow chart of the study selection process.

**Figure 2:** A forest plot of changes in V̇O_2_max for long-term and short-term training cessation. Mean and SD were reported on the plot and experimental group and control group means after detraining and before detraining, respectively. SMD: 95% confidence intervals (CI) and each study weight are shown on the right side. Gray boxes: each study's effect size, and gray diamonds: subgroup overall.

**Table 1:** Characteristics of the included studies.

Study	Training status	Duration (days)	Sample size (*n*)	Sex	Age	Cessation	Measures
Drinkwater et al. (1972) [27]	Lower	90	7	Female	<20	CDT	V̇O_2_max (ml/kg/min) HRmax (beats/min) Lactate (mEq/liter)
Murase, Y et al. (1981) [28]	Higher	730	5	Male	<20	CDT	V̇O_2_max (ml/kg/min)
Coyle et al. (1984) [29]	Higher	12, 21, 56, 84	7	Mixed	≥20	CDT	V̇O_2_max (ml/kg/min) HRmax (beats/min)
Cullinane et al. (1986) [30]	Higher	10	15	Male	≥20	CDT	V̇O_2_max (ml/kg/min) HRmax (beats/min)
Miyamura M et al. (1990) [31]	Lower	365, 455, 605, 730	5	Male	≥20	CDT	V̇O_2_max (ml/kg/min) HRmax (beats/min)
Houmard et al. (1992) [32]	Higher	14	12	Mixed	≥20	CDT	V̇O_2_max (ml/kg/min) HRmax (beats/min)
Madsen et al. (1993) [33]	Higher	28	9	Male	≥20	CDT	V̇O_2_max (l/min) HRmax (beats/min)
LaForgia et al. (1999) [34]	Lower	21	8	Male	≥20	CDT	V̇O_2_max (ml/kg/min)
Mochizuki et al. (1999) [35]	Higher	30	15	Mixed	<20	CDT	V̇O_2_max (ml/kg/min)
Doherty et al. (2003) [36]	Higher	15	7	Female	≥20	CDT	V̇O_2_max (ml/kg/min)
Petibois et al. (2003) [37]	Higher	35, 203, 364	10	Male	≥20	CDT	V̇O_2_max (ml/kg/min) Lactate (mEq/liter)
Gamelin et al. (2007) [38]	Lower	14,28, 56	14	Male	≥20	CDT	V̇O_2_max (ml/kg/min)
Caldwell et al. (2009) [39]	Lower	90	13	Male	≥20	PDT	V̇O_2_max (ml/kg/min)
J Garciapallares (2000) [40]	Higher	35	7	Male	≥20	CDT	V̇O_2_max (ml/kg/min) HRmax (beats/min) Lactate (mEq/liter)
Sotiropoulos et al. (2009) [41]	Higher	28	20,38	Male	≥20	PDT	V̇O_2_max (ml/kg/min)
Eastwood et al. (2012) [42]	Higher	30	9	Male	≥20	CDT	V̇O_2_max (ml/kg/min)
Koundourakis et al. (2014) [43]	Higher	42	23,22	Male	≥20	PDT	V̇O_2_max (ml/kg/min)
Koundourakis et al. (2014) [44]	Higher	42	67	Male	≥20	PDT	V̇O_2_max (ml/kg/min)
Melchiorri et al. (2014) [45]	Lower	42	14	Male	<20	CDT	V̇O_2_max (ml/kg/min) HRmax (beats/min)
Balague et al. (2016) [46]	Lower	21	8	Male	≥20	CDT	V̇O_2_max (ml/kg/min) HRmax (beats/min)
Melchiorri et al. (1999) [47]	Higher	56	15	Mixed	≥20	CDT	V̇O_2_max (ml/kg/min)

Duration (days): duration of detraining; higher: regular training will be conducted more than or equal to 5 times a week; lower: training will be less than 5 times a week; CDT: completely detraining; PDT: partly detraining.

The article "Effects of Short- and Long-Term Detraining on Maximal Oxygen Uptake in Athletes: A Systematic Review and Meta-Analysis" was published in 2022. Journal: Biomed Res Int.

**Table 2:** Strengthening the Reporting of Observational Studies in Epidemiology (STROBE).

Study	1	2	3	4	5	6	7	8	9	10	11	12	13	14	15	16	17	18	19	20	21	22	Overall
Murase et al.	1	2	2	2	1	1	2	2	0	0	2	0	1	2	2	2	0	2	1	2	1	0	28
Doherty et al.	2	2	2	2	1	1	2	2	1	0	2	2	2	2	2	2	0	2	2	2	2	1	36
Drinkwater et al.	1	2	2	2	1	1	2	1	0	0	2	2	1	2	2	2	0	2	1	2	1	0	29
Coyle et al.	1	2	2	2	1	1	2	2	1	0	2	2	1	2	2	2	2	2	1	2	1	2	35
Esatwood et al.	1	2	2	2	1	1	2	1	1	0	2	2	1	2	2	2	2	2	2	2	2	1	35
Houmard et al.	1	2	2	2	1	1	2	2	1	0	2	2	1	2	2	2	2	2	0	1	2	2	34
Yi-hung et al.	1	2	2	2	1	2	2	2	2	0	2	2	2	2	2	2	2	2	1	2	2	2	39
Petibois et al.	1	2	2	2	1	1	2	2	1	0	2	2	1	2	2	2	1	2	1	2	2	2	35
Balague et al.	1	2	2	2	1	1	2	2	1	0	2	2	2	1	2	2	2	2	2	2	2	2	37
Garcia et al.	2	2	2	2	1	1	2	2	0	0	2	2	2	2	2	2	0	2	2	2	1	1	34
LaForgia et al.	2	2	2	2	1	1	2	2	2	0	2	2	1	2	2	2	2	2	1	2	1	0	35
Mochizuki et al.	1	2	2	2	1	1	2	2	2	0	2	2	1	2	2	2	2	2	1	2	2	0	35
Androulakis et al.	1	2	2	2	1	2	2	2	2	0	2	2	2	2	2	2	2	2	2	2	2	1	39
TRAVLOS et al.	1	2	2	2	1	2	2	2	1	0	2	0	2	1	2	2	0	2	0	1	2	0	29
BRIAN et al.	1	2	2	2	1	1	2	1	2	0	2	0	2	1	2	2	0	2	2	2	2	1	32
Nikolaos et al.	1	2	2	2	1	2	2	2	2	0	2	0	2	1	2	2	0	2	2	2	2	1	34
Gamelin et al.	1	2	2	2	1	2	2	2	2	0	2	2	2	2	2	2	2	2	2	2	2	0	38
Eileen et al.	1	2	1	1	1	1	2	2	1	0	2	2	1	2	2	2	1	2	2	1	2	0	31
Melchiorri et al.	1	2	2	2	1	1	2	2	2	0	2	2	2	2	2	2	1	2	1	2	2	0	35
KLAVS et al.	1	2	2	2	1	1	2	2	1	0	2	1	1	2	2	2	2	2	1	2	1	1	33
Miharu et al.	1	2	2	2	1	1	2	2	1	0	2	0	1	2	2	1	2	0	1	2	2	1	30

1: title and abstract; 2: background/rationale; 3: objectives; 4: study design; 5: setting; 6: participants; 7: variables; 8: data sources/measurement; 9: bias; 10: study size; 11: quantitative variables; 12: statistical methods; 13: participants; 14: descriptive data; 15: outcome data; 16: main results; 17: other analyses; 18: key results; 19: limitations; 20: interpretation; 21: generalizability; and 22: funding (0: no information; 1: low; and 2: high).

The article "Effects of Short- and Long-Term Detraining on Maximal Oxygen Uptake in Athletes: A Systematic Review and Meta-Analysis" was published in 2022. Journal: Biomed Res Int.

**Table 3:** Subgroup analysis of the long-term detraining effect on V̇O_2_max.

	*k*	SMD	95% CI	*p*	*Q*	*I* ^2^
Duration						
30-90 days	12	-1.6	-2.47; -0.74	<0.001	64.36	0.83
>90 days	7	-1.20	-2.13; -0.28	<0.001	14.66	0.59
Training state						
Higher	10	-1.91	-2.57; -1.25	<0.001	28.8	0.69
Lower	4	-0.85	-1.83; 0.12	<0.001	24.5	0.67
Age						
<20^b^	3	-2.81	-6.32; 0.69	<0.001	5.04	0.63
≥20	16	-1.20	-1.76; -0.64	<0.001	58.4	0.74
Format						
CDT	16	-1.69	-2.41; -0.96	<0.001	52.5	0.73
PDT	4	-0.65	-1.42; 0.11	<0.001	9.2	0.67

*k*: number of studies; SMD: <-0.5, small; 0.5 to 0.8, moderate; and >0.8, large; *I*^2^: heterogeneity test.

**Table 4:** Subgroup analysis of the short-term detraining effect on V̇O_2_max.

	*k*	SMD	95% CI	*p*	*Q*	*I* ^2^
Training status						
Higher	7	-0.76	-1.10; -0.41	<0.001	9.32	0.37
Lower	7	-0.46	-0.75; -0.18	0.014	9.39	0.36
Age						
<20	1	-0.83	-1.57; -0.08	0.030	—	—
≥20	13	-0.61	-0.95; -0.26	<0.001	19.3	0.38
CDT	11	-0.54	-0.82; -0.26	<0.001	14.4	0.31
PDT	3	-0.65	-1.00; -0.30	0.01	5.76	0.65

*k*: number of studies; SMD: <-0.5, small; 0.5 to 0.8, moderate; and >0.8, large; *I*^2^: heterogeneity test.

## Data Availability

The data used to support the findings of this study are included within the article.
